# Isoalantolactone inhibits IKKβ kinase activity to interrupt the NF‐κB/COX‐2‐mediated signaling cascade and induces apoptosis regulated by the mitochondrial translocation of cofilin in glioblastoma

**DOI:** 10.1002/cam4.2013

**Published:** 2019-02-10

**Authors:** Jin‐Shan Xing, Xun Wang, Yu‐Long Lan, Jia‐Cheng Lou, Binbin Ma, Tingzhun Zhu, Hongqiang Zhang, Dongsheng Wang, Zhikuan Yu, Zhongbo Yuan, Xin‐Yu Li, Bo Zhang

**Affiliations:** ^1^ Department of Neurosurgery The Second Affiliated Hospital of Dalian Medical University Dalian China; ^2^ Department of Neurosurgery Shenzhen People's Hospital Shenzhen China; ^3^ Department of Neurosurgery The Third People's Hospital of Dalian Non‐Directly Affiliated Hospital of Dalian Medical University Dalian China; ^4^ Department of Endocrinology Dalian Municipal Central Hospital Affiliated of Dalian Medical University Dalian China

**Keywords:** cofilin, COX‐2, glioblastoma, IATL, NF‐κB

## Abstract

Isoalantolactone (IATL), a sesquiterpene lactone compound, possesses many pharmacological and biological activities, but its role in glioblastoma (GBM) treatment is still unknown. The aim of the current study was to investigate the antiglioma effects of IATL and to explore the underlying molecular mechanisms. In the current study, the biological functions of IATL were examined by MTT, cell migration, colony formation, and cell apoptosis assays. Confocal immunofluorescence techniques, chromatin immunoprecipitation, and pull‐down assays were used to explore the precise underlying molecular mechanisms. To examine IATL activity and the molecular mechanisms by which it inhibits glioma growth in vivo, we used a xenograft tumor mouse model. Furthermore, Western blotting was used to confirm the changes in protein expression after IATL treatment. According to the results, IATL inhibited IKKβ phosphorylation, thus inhibiting both the binding of NF‐κB to the cyclooxygenase 2 (COX‐2) promoter and the recruitment of p300 and eventually inhibiting COX‐2 expression. In addition, IATL induced glioma cell apoptosis by promoting the conversion of F‐actin to G‐actin, which in turn activates the cytochrome c (Cyt c) and caspase‐dependent apoptotic pathways. In the animal experiments, IATL reduced the size and weight of glioma tumors in xenograft mice and inhibited the expression of COX‐2 and phosphorylated NF‐κB p65 in the transplanted tumors. In conclusion, the current study indicated that IATL inhibited the expression of COX‐2 through the NF‐κB signaling pathway and induced the apoptosis of glioma cells by increasing actin transformation. These results suggested that IATL could be greatly effective in GBM treatment.

## 1 INTRODUCTION

Glioblastoma (GBM) is the most common primary tumor of the central nervous system (CNS).^1^ The current treatment strategy for GBM is mainly comprised of surgical approaches combined with radiotherapy and chemotherapy. However, achieving complete resection is difficult because most GBMs are characterized by invasive growth without clear boundaries with the surrounding normal brain tissue.^2^ In addition, GBM is usually not sensitive to radiotherapy and chemotherapy, and unfortunately, these treatments do not significantly improve the median survival of patients.^3^ Thus, the identification of a drug that can penetrate the blood‐brain barrier (BBB) and target GBM cells specifically^4^ will prolong the survival of GBM patients and improve their quality of life.

Experiments have shown that inflammation increases the risk of cancer.^5^, ^6^, ^7^, ^8^ Inflammatory factors in the microenvironment could be greatly associated with tumor migration, viability, invasion, etc.^9^, ^10^, ^11^; thus, inhibitors of inflammation can play an important role in the treatment of malignant tumors. Cyclooxygenase 2 (COX‐2) has been demonstrated to have an important effect in mediating inflammation.^9^, ^10^, ^11^, ^12^ COX‐2‐selective inhibitors can inhibit the inflammatory response, cell proliferation, and angiogenesis and can induce cancer cell apoptosis. Previous studies have indicated that the overexpression of COX‐2 in glioma cells could affect the development of glioma, and an increase in COX‐2 expression is also associated with the histopathological grade and invasiveness of glioma, which ultimately lead to poor prognoses for patients.^13^, ^14^, ^15^, ^16^, ^17^ In general, reducing the expression of COX‐2 may be an effective alternative to inhibit glioma growth and promote apoptosis.

The expression of COX‐2 is regulated by various *trans* factors, such as NF‐κB, transcriptional coactivator p300 and p65, which bind to the corresponding promoter region to regulate transcription.^18^, ^19^, ^20^, ^21^ The overexpression of COX‐2 is related to the activation of the NF‐κB signaling pathway.^22^, ^23^ The activation of the NF‐κB signaling pathway is mediated by the degradation of IκB, and the IκB kinase (IKK) complex can rapidly phosphorylate IκB. The IKK complex is composed of the IKKα and IKKβ catalytic subunits, in which IKKβ has the more important role in the phosphorylation of the IκB protein; its regulatory subunit is IKKγ/NF‐κB essential regulator (NEMO).^24^ The subsequently phosphorylated IκB is degraded by proteasomes to release free NF‐κB dimers, which are further translocated to the nucleus for gene transcription.^25^ Thus, finding a small molecule inhibitor that targets and inhibits IKKβ to regulate NF‐κB activation is important.

Isoalantolactone (IATL), a sesquiterpene lactone compound purified from the roots of *Inula helenium* L., has long been used in Chinese traditional medicine.^26^ IATL exert a desirable effect and does not cause serious injury to normal tissue. Experiments have shown that IATL can induce a highly selective cytotoxic effect, while its toxicity to the body's normal peripheral blood lymphocytes is very low.^27^ The antitumor properties of IATL in lung and breast cancers have already been reported.^28^, ^29^, ^30^ However, the effects of IATL in GBM have not yet been confirmed.

In the current study, the inhibitory effect of IATL in GBM was explored via in vivo and in vitro experiments. In addition, the molecular mechanisms by which IATL inhibits GBM were investigated by detecting changes in the NF‐κB signaling pathway (as well as in cofilin, F‐actin, and G‐actin). Finally, we measured the IATL level in the cerebrospinal fluid in the nude mouse model, confirming that IATL could penetrate the BBB. In summary, IATL has great potential as a new strategy for the treatment of CNS tumors.

## 2 MATERIALS AND METHODS

### 2.1 Drugs and reagents

Isoflavone (IATL) was prepared by our laboratory; the purity was ≥98.7% (measured by HPLC and compared with standard reference), and the structure was identified by ^1^H‐NMR and ^13^C‐NMR. Extraction and purification were performed via stepwise elution in a solvent system containing n‐hexane:ethyl acetate:methanol:water in volumetric ratios of 4:6:2:4, 4:6:2.5:4, and 4:6:3.2:4. The concentration of the parenteral lactone mother liquor was 100 μmol/L. The mother liquor was dissolved in dimethyl sulfoxide (DMSO) and stored at −20°C, and the final concentration of DMSO was <0.1% when applied to cells. RPMI 1640 medium and DMEM were purchased from HyClone, Northbrook, IL, USA; streptomycin was purchased from HyClone; premium fetal calf serum was purchased from Israel Biological Industries (Kibbutz Beit Haemek, Israel); 0.25% trypsin‐EDTA was purchased from Beijing Suobao Technology Co., Ltd. (Beijing, China); and MTT, DMSO, and streptavidin‐agarose were purchased from Sigma (St. Louis, MO, USA).

An Annexin V‐FITC Apoptosis Detection kit was purchased from Nanjing Kaiji Biotechnology (Nanjing, Jiangsu, China); Protein A/G PLUS‐Agarose was purchased from Changchun Jitai Yuancheng (Changchun, Jilin, China); a BCA protein quantification kit was purchased from Beijing Kangwei Century (Beijing, China); mammalian protein extraction reagent was purchased from Beijing Kangwei Century; an SP immunohistochemistry kit was purchased from Jinshan Jinqiao (Beijing, China); anti‐COX‐2, anti‐IKKα, anti‐IKKβ, anti‐p‐IKKα/β, and anti‐NF‐κB p65/p‐p65 antibodies were purchased from Cell Signaling Technology (Pudong, Shanghai, China). All other chemicals were purchased from Sigma unless otherwise specified.

### 2.2 Cell culture

Human U87MG, U251, U118, and SHSY‐5Y cell lines were obtained from the American Type Culture Collection (ATCC, Manassas, VA, USA). All cells were maintained in DMEM supplemented with 10% fetal bovine serum (FBS) at 37°C in a humidified atmosphere containing 5% CO_2_.

### 2.3 Determination of cell viability by the MTT assay

U251 and U87 cells in the logarithmic growth phase were trypsinized to make a single‐cell suspension of 6 × 10^4^ cells/mL, and 100 μL per well of this suspension was inoculated in 96‐well plates and maintained in a CO_2_ incubator. After incubation for 24 hours, cell growth was observed under a microscope. If the growth was appropriate, the original cell culture medium was aspirated, and fresh medium containing different concentrations of the drug solution (0, 10, or 20 μmol/L IATL) was added. A blank control group and a 0.1% DMSO control group were set up, for a total of five groups. Two wells per condition were cultured in a CO_2_ incubator. After the cells were incubated for 48 hours, the original cell culture medium was aspirated, and blank (serum‐free) medium containing a final concentration of 0.5 mg/mL MTT was added. The cells were cultured for a further 4 hours, and the supernatant was discarded. Then, 150 μL DMSO was added with shaking for 10 minutes, and the absorbance was measured at 490 nm using a multifunction microplate reader. Cell viability was calculated with the following formula: Cellular viability (%) = [(treated) OD − (blank) OD]/[(0.1% DMSO) OD − (blank) OD] × 100. A column chart showing the cell proliferation activity was generated with the cell viability as the ordinate and the drug concentration as the abscissa.

### 2.4 Transwell invasion assay

Cell invasion was analyzed using a Transwell assay. U87 and U251 cells were plated in 24‐well Transwell plates. The upper surface of the polycarbonate filters was coated with Matrigel and incubated for 1 hour at 37°C for gelling. The cells (5 × 10^4^) were seeded into the upper chambers in FBS‐free DMEM, and the bottom chambers were filled with 600 μL of DMEM supplemented with 10% FBS. Both the top and bottom chambers contained the same concentrations of IATL. After 24 hours of incubation, the noninvasive cells on the upper membrane surfaces were removed by wiping with cotton swabs. The invading cells were fixed with methanol and stained with a 0.1% crystal violet staining solution. Images were acquired under a Leica DM 14000B microscope. Cell invasion was counted in five independent areas per membrane. The results are represented as the means calculated from five replicates of each experiment.

### 2.5 Flow cytometry analysis

To determine the distribution of the cells in the cell cycle and the proportion of apoptotic cells, we performed a flow cytometry analysis using a flow cytometer (BD FACS Accuri C6, Shanghai, China). After treatment with IATL (0, 10, and 20 μmol/L) for 24 hours, the cells were collected, washed with PBS, and fixed with ice‐cold 70% ethanol at 4°C for 4 hours. The cells were stained with propidium iodide (PI) staining buffer (0.2% Triton X‐100, 100 μg/mL DNase‐free RNase A, and 50 μg/mL PI in PBS) in the dark for 30 minutes. For the apoptosis examination, the cells were washed with PBS, collected, and stained using an Annexin V‐FITC Apoptosis Detection kit in the dark at room temperature for 15 minutes. The cell cycle distribution and the fraction of apoptotic cells were determined using a fluorescence‐assisted cell sorting (FACS) analysis system. Each experiment was performed in triplicate.

### 2.6 Western blot analysis

The cell lysate proteins were separated by electrophoresison a 7.5%‐12% SDS‐PAGE and probed with specific antibodies. The protein bands were detected by enhanced chemiluminescence. The protein concentrations were determined using a BCA protein assay kit (Beyotime Biotechnology, Shanghai, China). Similar experiments were performed at least three times.

### 2.7 Reverse‐transcriptase polymerase chain reaction (RT‐PCR)

Total RNA was extracted from ATL‐treated U87 and U251 cells using the TRIzol reagent, according to the kitprotocol (TaKaRa Bio, Dalian, China). The cDNA was reverse‐transcribed using the Prime Script RT Reagent kit (TaKaRa Bio), according to the manufacturer's instructions. The primer pairs were as follows: COX‐2, Forward: 5′‐TCACAGGCTTCCATTGACCAG‐3′ and Reverse: 5′‐CCGAGGCTTTTCTA CCAGA‐3′; β‐actin, Forward: 5′‐GGCACCCAGCACAATGAA‐3′ and Reverse: 5′‐TAGAAGCATTTGCGGTGG‐3′. The amplification products were analyzed using a 1.5% agarose gel electrophoresis, stained with ethidium bromide, and photographed under ultraviolet light.

### 2.8 Confocal immunofluorescence

Briefly, IATL‐treated U87 cells were grown on chamber slides, fixed with 4% paraformaldehyde and permeabilized with 0.2% Triton X‐100. The samples were probed with specific antibodies against cytochrome c (Cyt c), p300, p50, or p65 (Santa Cruz) and then with fluorescein isothiocyanate‐ and rhodamine‐conjugated secondary antibodies. Subsequently, the cell nuclei in the stained samples were counterstained with 4′,6‐diamidino‐2‐phenylindole. After five additional 5‐minute washes, the samples were examined under a Leica DMI 4000B confocal microscope.^31^

For the observation of F‐actin/G‐actin conversion via laser confocal microscopy, U87 cells were resuspended to a concentration of 3.5 × 10^5^ cells/mL and inoculated in 24‐well plates at 1 mL/well. The cells were incubated for 24 hours, and 30 μmol/L IATL was added, and incubation was continued for 48 hours, at which time the cells were collected by centrifugation and washed twice with PBS, and the plate was placed on a glass slide. A single cell was collected, and the cells were allowed to dry. The slide was placed into ice‐cold acetone and fixed at room temperature for 30 minutes. The slide was then washed 10 times with PBS for 3 minutes each, washed one time with 0.1% Triton X‐100 for 10 minutes, washed three times with PBS for 10 minutes each, blocked with normal goat serum working fluid for 30 minutes, and rinsed three times with PBS. Fluorescent phallotoxins diluted 1:40 and fluorescent deoxyribonuclease I diluted 1:500 were added dropwise to the slides, which were then incubated at 37°C for 30 minutes, rinsed two times with PBS, washed three times for 10 minutes each, and mounted in 70% glycerol for confocal observation. Images were then acquired.

To examine the colocalization of cofilin, F‐actin, G‐actin, and mitochondria, U87 cells were inoculated at a volume of 1 mL/well into 24‐well plates at 0.5 × 10^5^ cells/minute and incubated in an incubator. After 24 hours, 30 μmol/L IATL was added, and incubation was continued for 24 hours, at which time the cells were incubated with Mito Tracker Red CMXRos (500 nmol/L) for 30 minutes, centrifuged for 5 minutes at 800 rpm and 4°C, and washed twice with PBS. The cells were deposited on the slide to produce a single‐cell dispersion. The slide was air‐dried, placed into ice‐cold acetone, fixed at room temperature for 30 minutes, and air‐dried after immunostaining. The cells were washed 10 times with PBS for 3 minutes each, washed one time with 0.1% Triton X‐100 for 10 minutes, washed three times with PBS for 10 minutes each, blocked with normal goat serum working fluid for 30 minutes, rinsed three times with PBS, and incubated with fluorescent phallotoxins (1:40) and fluorescent deoxyribonuclease I (1:500). The cofilin antibody was diluted 1:50 and then added to different groups of cells. After incubation at 37°C for 1 hour, the cells were incubated overnight at 4°C. The slides were then washed for 10 minutes each, and an Alexa Fluor 488‐conjugated goat anti‐mouse secondary antibody diluted 1:300 was added dropwise to the target cells for immunofluorescence staining. The cells were incubated at 37°C for 1 hour, rinsed two times in PBS, washed three times for 10 minutes each, and mounted in 70% glycerol for confocal observation. Images were then acquired.

### 2.9 Streptavidin‐agarose pull‐down assay to detect DNA protein binding

The binding assay was performed by mixing 400 μg of the nuclear extract proteins, 4 μg of the biotinylated DNA probe, and 40 μL of 4% streptavidin‐conjugated agarose beads at RT for 5 hours in a rotating shaker. The beads were centrifuged, resuspended with the SDS‐PAGE loading buffer, and boiled at 95°C. The supernatant was analyzed by Western blotting.

### 2.10 Chromatin immunoprecipitation (ChIP)

The ChIP assay was performed as previously described.^32^ The specific COX‐2 promoter primers were as follows: forward primer: ACGTGACTTCCTCGACCCTC, and reverse primer: AAGACTGAAAA CCAAGCCCA. The resulting 478 bp product of COX‐2 was separated by 1.5% agarose gel electrophoresis.

### 2.11 IKKβ kinase activity assay in vitro

IATL‐mediated inhibition of IKKβ kinase activity was assessed in vitro using a cell IKKβ kinase activity spectrophotometry quantitative detection kit. Briefly, IATL‐treated U87 cells were harvested and lysed with the lysate in the kit. After the protein was quantified, 10 μL of the sample solution (containing 50 μg of protein) was mixed with the reaction solution in the kit. The total activity and nonspecific activity were measured using a microplate reader. The data were evaluated according to the formula in the manual, and the specific activity value was calculated (specific activity = total activity‐nonspecific activity).

### 2.12 Animal studies

Male nude mice (BALB/c nu/nu, 4 weeks old, 18‐19 g) were purchased from the SPF Laboratory Animal Center of Dalian Medical University (Dalian, China). Briefly, 1 × 10^7^ U87 cells were injected subcutaneously near the axillary fossa of the nude mice. The tumor cell‐inoculated mice were randomly divided into the following two treatment groups with five mice in each group: group A was treated with propylene glycol; group B was treated with 30 mg/kg IATL; all treatments were delivered by daily intraperitoneal injections. The tumors were measured using a caliper every 2 days, and the tumor volume was calculated according to the formula *V* = 1/2 (width [2] × length). The body weights were also recorded. After treatment with IATL for 15 days, all experimental mice were terminated with ether anesthesia, and the total weight of the tumors in each mouse was measured. To determine the expression of COX‐2 and NF‐κB p65, the tumor tissues were fixed with 10% neutral formalin and embedded in paraffin. The sections (4 μm) were stained with the COX‐2 antibody (1:50) and the p‐p65 NF‐κB (1:50) antibody and examined under a light microscope. The images were examined under a Leica DM 4000B microscope equipped with a digital camera.

All animals were given free access to sterilized food and water and were habituated for 7 days before the experiments. All procedures were in accordance with the National Institutes of Health Guide for the Care and Use of Laboratory Animals (National Institutes of Health, Bethesda, MD, USA). The protocol was approved by the Animal Care and Ethics Committee of Dalian Medical University.

### 2.13 Detection of IATL through the BBB

Six male adult SD rats (200‐220 g) were intraperitoneally injected with IATL; after 1 hour, the rats were anesthetized with 4% chloral hydrate. Cerebrospinal fluid (50‐100 μL) was collected from the cerebellomedullary cistern by puncturing the foramen magnum. Then, the cerebrospinal fluid was extracted twice using an equal volume of acetonitrile. The supernatant was dried in a nitrogen blowing instrument and reconstituted in 50 μL mobile phase (acetonitrile:pure water = 45:55). Finally, their constituted sample and IATL standard solution were analyzed by LC‐MS/MS.

### 2.14 Statistical analysis

Student's *t* test (two‐tailed), *t* test with Welch's correction, *F* test were performed to analyze the data using GraphPad Prism 6.0 software (GraphPad software, Inc., La Jolla, CA, USA). The concrete methods of *t* test analysis in current study are as follows: The data of two groups for comparison were analyzed by *F* test firstly (homogeneity test of variance): If the value of *F* test >0.05, the value of *t* test was obtained according to heteroscedasticity double sample test. If the value of *F* test <0.05, the value of *t* test was obtained according to the heteroscedasticity double sample test; The value of *t* test <0.05 indicated that there was significant difference between the two experimental groups, and the value of *t* test >0.05 indicated that there was no significant difference between the two experimental groups. Two‐way analysis of variance (ANOVA), followed by a Bonferroni's test for multiple comparisons, were performed to analyze the data for Figures 1c, 5e,f, 6c, 7c, and 8c. While one‐way ANOVA, followed by a Tukey's posttest for multiple comparisons, were performed to analyze the data for Figure 2b. The data are represented as the mean ± SD of at least three independent experiments. *P* < 0.05 was considered statistically significant. SPSS18.0 software (SPSS Inc., Chicago, IL, USA) was used for all statistical analyses.

**Figure 1:** Isoalantolactone (IATL) changed cell morphology and inhibited cancer cell viability. A, Chemical structure of IATL. B, Changes in the morphology and proliferation of U87 and U251 cells after IATL treatment for 48 h. C, MTT assays were performed after incubation with the indicated concentrations of IATL for the indicated times. D, Cell viability was measured using the MTT assay after treatment with IATL for 48 h and was followed by the calculation of the IC_50_ values. *P < 0.05, **P < 0.01 vs the dimethyl sulfoxide‐treated group

**Figure 2:** Isoalantolactone (IATL) inhibited cell colony formation and blocked the cell cycle. A, Glioma cells were treated with IATL at the indicated doses, the induced colony formation was analyzed, and the number of colonies formed was calculated. B, Cell cycle analysis was performed after IATL treatment for 48 h. C, The levels of the cell cycle‐related proteins cyclin D and CDK4 in U87 cells in the G1 phase of the cell cycle were assessed by Western blotting. The data are presented as the means ± SDs of three independent experiments (*P < 0.05, **P < 0.01; significant differences between IATL‐treated and dimethyl sulfoxide vehicle controls)

## 3 RESULTS

### 3.1 IATL suppressed cell viability and altered cell morphology in human GBM cells

The inhibition of cell viability could be important for cancer treatment.^33^ First, the effects of various concentrations (1, 10, 25, and 50 μmol/L) of IATL on cell proliferation were examined in several GBM cell lines (Figure 1a) for 24, 48, and 72 hours. As shown in Figure 1b,c, IATL significantly inhibited the proliferation of the cancer cells (U118, U87, U251, and SH‐SY5Y cells) in a dose‐ and time‐dependent manner. The IC_50_ values of IATL for inhibiting cell viability in the four cell lines were also calculated and found to be 30.26 ± 2.11 μmol/L (U87), 32.57 ± 1.93 μmol/L (U251), 33.17 ± 2.84 μmol/L (U118), and 26.12 ± 2.38 μmol/L (SH‐SY5Y) (Figure 1b). Furthermore, the effect of IATL on cell morphological changes in human U87 and U251 GBM cells was also assessed. As shown in Figure 1d, IATL reduced cell‐to‐cell contact, and treated cells exhibited less spreading with less formation of filopodia than did the control groups. These results demonstrated that IATL exhibited potential antitumor activity in GBM.

### 3.2 IATL promoted cell colony formation inhibition and cell cycle arrest

The clonal and proliferative capacity of tumor cells is a key factor in pathogenesis. Thus, a colony formation experiment was used to evaluate the effect of IATL on the colony‐forming ability of U87 and U251 cells. As shown in Figure 2a, IATL significantly inhibited colony formation and reduced the number of colonies formed. Cell proliferation inhibition is associated with cell cycle arrest^34^; therefore, we next evaluated the degree to which IATL affects cell cycle arrest. As shown in Figure 2b, a substantial proportion of IATL‐treated cells exhibited growth arrest at the G0/G1 phase, and the effect was dose‐dependent. The percentage of cells in the G0/G1 phase increased from 61.15% to 76.75%; on the contrary, the percentage of cells in the S and G2/M phases decreased from 26.56% to 19.48% and from 13.21% to 7.27%, respectively (Figure 2b). Furthermore, we examined the expression of several cell cycle‐related proteins, including cyclin D and CDK4, in the U87 cells after treatment with IATL for 48 hours. The results showed that treatment with IATL resulted in a dramatic reduction in the expression of these proteins (Figure 2c). These data provide evidence that IATL could induce the inhibition of cell proliferation at least in part by inducing cell cycle arrest at the G0/G1 phase.

### 3.3 IATL suppressed the migratory ability of GBM cells

Wound healing assays and Transwell assays were employed to detect the effect of IATL on the migratory ability of GBM cells. As shown in Figure 3a,b, treatment with IATL significantly inhibited the migration and invasion of GBM cells. In addition, we also assessed the expression of key protein markers associated with cell migration and invasion, including matrix metalloproteinases (MMPs) and found that IATL significantly inhibited the expression of MMP‐2 and MMP‐9 (Figure 3c). Therefore, IATL showed a strong inhibitory effect on the migration and invasion of GBM cells.

**Figure 3:** Isoalantolactone (IATL) inhibited cancer cell migration and cell invasion. A, The migration of glioma cells was tested using the wound healing assay. B, The inhibitory effect of IATL on cell invasion was examined by using Transwell assays. U87 cells were placed in Matrigel‐precoated Transwell chambers. Cells crossing the membrane were counted (original magnification, 100 × ). C, The expression of the invasion markers matrix metalloproteinase 2 (MMP‐2) and MMP‐9 was detected by Western blotting. *P < 0.05, **P < 0.01 vs the dimethyl sulfoxide‐treated group

### 3.4 IATL induced the dedifferentiation of filamentous F‐actin into globular G‐actin monomers and the translocation of cofilin and G‐actin to mitochondria

The U87 glioma cells were treated with IATL, and mitochondrial proteins, cytoplasmic proteins, and whole‐cell proteins were extracted. IATL induced a gradient of cofilin expression in the cytoplasmic fraction of U87 cells by gradually increasing cofilin expression in the mitochondrial fraction; however, the expression of cofilin in the whole‐cell lysate did not change significantly, suggesting that IATL induced dose‐dependent translocation of the cofilin protein from the cytoplasm to the mitochondria. However, although the expression of the whole‐cell and cytosolic p‐cofilin (Ser 3) protein was downregulated, no p‐cofilin (Ser 3) band was seen in the mitochondrial fraction, suggesting that the phosphorylation of cofilin cannot lead to its mitochondrial translocation (Figure 4a).

**Figure 4:** Isoalantolactone (IATL) induced filamentous F‐actin depolymerization into globular G‐actin monomers and promoted the mitochondrial translocation of G‐actin and cofilin. A, Assessment of intracellular and mitochondrial cofilin and actin by Western blot analysis. B, Assessment of F‐actin and G‐actin by Western blot analysis. C, The conversion of F‐actin to G‐actin was observed by immunofluorescence confocal analysis. D and E, The relationship between F‐actin, G‐actin, cofilin, and mitochondria was examined by immunofluorescence confocal analysis. F, The direct binding of cofilin to actin was detected by immunoprecipitation. The results are expressed as the means ± SDs of three independent experiments. (**P < 0.05, **P < 0.01 vs the dimethyl sulfoxide‐treated group)

After the treatment of U87 cells with the indicated dose of IATL, G‐actin and F‐actin were isolated by the G‐actin/F‐actin isolation kit. The results of Western blotting showed an increase in both F‐actin and G‐actin (Figure 4b). Staining of F‐actin and G‐actin was investigated by immunofluorescence confocal microscopy; the fluorescence from F‐actin was downregulated and the fluorescence from G‐actin was increased (Figure 4c). From this result, it can be speculated that G‐actin is transferred to mitochondrial actin. To validate this hypothesis, immunofluorescence confocal experiments, immunofluorescence staining of cofilin proteins, and dye staining of G‐actin and mitochondria were further used. IATL has also been shown to promote the colocalization of cofilin and G‐actin (Figure 4d). To further verify the distribution of F‐actin and G‐actin in the mitochondria and cytoplasm, we performed immunofluorescence confocal experiments in U87 cells treated with the indicated dose of IATL. In the mitochondria of the experimental group, the level of G‐actin protein increased and that of F‐actin decreased (Figure 4e). Furthermore, the mitochondrial, cytoplasmic, and whole‐cell fractions were extracted from U87 cells after IATL treatment, and immunoprecipitation techniques were used to detect the direct binding of cofilin to G‐actin. The results showed that IATL increased the direct binding of cofilin and G‐actin in the mitochondrial fraction (Figure 4f). The results of the Western blot analysis were thus confirmed. Taken together, the results of these two experiments show that IATL induces the mitochondrial translocation of cofilin and G‐actin and directly increases the mitochondrial content of cofilin and actin, in turn leading to mitochondrial damage.

### 3.5 Cofilin and G‐actin translocated to mitochondria to induce apoptosis through regulating Cyt c and caspase signaling

Apoptosis is a cell suicide mechanism, and the induction of apoptosis is a key mechanism underlying anticancer therapy.^35^, ^36^ According to the literature, the release of Cyt c from mitochondria to the cytoplasm is a key step in the activation of apoptosis.^37^ We thus examined whether the IATL‐induced inhibition of cell growth is associated with increased apoptosis of neuroblastoma cells. IATL treatment resulted in significant dose‐dependent induction of apoptosis in U87 cells (Figure 5a). After the treatment of U87 cells with a concentration gradient of IATL, the expression of Cyt c increased in the cytoplasm, as determined by Western blotting (Figure 5b). In addition, changes in the localization of Cyt c in U87 cells were examined by immunofluorescence imaging, and Cyt c was found to be strongly released from the mitochondria into the cytoplasm after the treatment of the cells with IATL (Figure 5c). For further validation, we performed Western blot assays to detect the expression of three key proapoptotic proteins (PARP, caspase‐3, and caspase‐9) and of BAX and Bcl‐2. Treatment with IATL significantly increased the expression of cleaved caspase‐3/‐9, cleaved PARP, and BAX protein and decreased the level of Bcl‐2 protein (Figure 5d). The above results indicate that IATL eventually leads to the release of Cyt c from the mitochondria, triggering apoptosis. Furthermore, a decreased oxygen consumption rate was induced by IATL (Figure 5e). JC‐1 (a fluorescent probe used to test the mitochondrial membrane potential) staining indicated that increased cell death was inversely correlated with decreased mitochondrial membrane potential in IATL‐treated cells. IATL treatment decreased the mitochondrial membrane potential, as detected by the enhanced intensity of the green fluorescence signal and the reduced intensity of the red JC‐1 fluorescence signal (Figure 5f).

**Figure 5:** Isoalantolactone (IATL) induced apoptosis by regulating cytochrome c (Cyt c)/caspase signaling. A, Detection of the expression of the indicated apoptosis‐related proteins by Western blot analysis. B, By using immunofluorescence imaging analysis in U87 cells, the release of Cyt c from mitochondria into the cytoplasm was examined. C, Apoptosis was assessed using FACS. All data are presented as the means ± SDs of three independent experiments. *P < 0.05, **P < 0.01 vs the dimethyl sulfoxide (DMSO)‐treated group. D, The cytoplasmic protein expression of Cyt c was examined by using Western blotting. E, IATL induced a reduction in the oxygen consumption rate. F, U87 cells were exposed to the indicated doses of IATL for 24 h. Changes in the mitochondrial membrane potential were determined by JC‐1 staining, and a quantitative analysis of the shift of mitochondrial orange‐red fluorescence to green fluorescence in the groups (red/green fluorescence ratio) was conducted. Data from three independent experiments are shown. The results are expressed as the means ± SDs of three independent experiments. *P < 0.05, **P < 0.01 vs the DMSO‐treated group

### 3.6 IATL suppressed COX‐2 signaling in human GBM cells

Studies have shown that the growth, migration, and invasion of cancer cells are associated with high expression of COX‐2.^32^, ^38^, ^39^, ^40^ To investigate whether IATL affects the COX‐2 signaling pathway in GBM, Western blotting and RT‐PCR were performed to analyze the protein and gene expression of COX‐2. First, COX‐2 expression was evaluated in CNS tumor cell lines, including U118, SHSY‐5Y, U251, and U87. As shown in Figure 6a, the expression of COX‐2 was more abundant in U251 and U87 cells than in the other cell lines. We next evaluated the effect of IATL on COX‐2 expression in U251 and U87 cells. The results showed that treatment with IATL significantly decreased COX‐2 expression at both the protein and mRNA levels (Figure 6b). Furthermore, U87 cells were pretreated with the COX‐2‐selective inhibitor celecoxib (CB, 60 and 120 μmol/L) for 8 hours and then treated with IATL for another 48 hours. Cell viability was analyzed by a CCK‐8 assay. As shown in Figure 6c, treatment with CB or IATL alone resulted in different inhibitory effects on cell viability, whereas the combined treatment did not significantly alter the inhibition of cell viability. The above results implied that the inhibitory effect of IATL on the proliferation of GBM cells is partially mediated by inactivated COX‐2 signaling.

**Figure 6:** Isoalantolactone (IATL) inhibited cyclooxygenase 2 (COX‐2) expression. A, The expression of COX‐2 in four neural tumor cell lines was assessed by using Western blot analysis. B, The expression of COX‐2 protein and mRNA after treatment with IATL for 48 h were examined by Western blotting and RT‐PCR, respectively. C, U87 cells were pretreated with the COX‐2‐selective inhibitor CB (60 and 120 μmol/L) for 8 h and were then treated with IATL (30 μmol/L). Forty‐eight hours later, cell viability was assessed using the MTT assay. All data are expressed as the means ± SDs of three independent experiments (*P < 0.05, **P < 0.01 vs the dimethyl sulfoxide vehicle control group). (D‐G) In addition, the inhibitory effects of IATL on the translocation of NF‐κB p65/p50 and p300 and the binding of these proteins to the COX‐2 promoter were explored. D, After IATL treatment for 48 h, the binding of p300, p65, and p50 to the COX‐2 promoter probe in glioma cells was examined by the streptavidin‐agarose pull‐down assay. E, Chromatin was immunoprecipitated with anti‐p50, anti‐p65, and anti‐p300 antibodies 48 h after IATL treatment; the level of the COX‐2 promoter region in the precipitated chromatin was then determined by RT‐PCR. F, Cytoplasmic and nuclear proteins were first isolated, and p65 and p50 expression was then assessed by using Western blot analysis. G, The subcellular localization of p65, p50, and p300 and the colocalization of p50 with p65 or p300 were assessed by confocal microscopy

### 3.7 IATL abrogated the translocation of NF‐κB and p300 and the binding of these proteins to the COX‐2 promoter

Studies have shown that the transcription factor NF‐κB and the transcriptional coactivator p300 are involved in the regulation of COX‐2 expression.^41^ Thus, by using a 478‐bp biotin‐labeled double‐stranded oligonucleotide probe, we carried out a streptavidin‐agarose pull‐down assay to examine the effect of IATL on the binding activities of NF‐κB and p300 to the COX‐2 promoter (nucleotide positions ‐30 to ‐508). The results showed that compared with the control treatment, treatment with IATL significantly suppressed the binding of the NF‐κB p50/p65 subunits and p300 to the COX‐2 promoter DNA probe (Figure 6d) in a dose‐dependent manner. To further confirm these results, a ChIP assay using specific antibodies was performed. As shown in Figure 6e, IATL also markedly suppressed the binding of NF‐κB p50/p65 and p300 to the COX‐2 promoter in chromatin. Subsequently, we assessed the subcellular distribution of the NF‐κB p50/p65 subunits after treatment with IATL. As shown in Figure 6f, IATL significantly reduced the protein levels of p65/p50 in the nucleus; however, IATL had no obvious effects on the expression of these proteins in the cytoplasm in U87 and U251 cells. Based on the above results, we hypothesized that IATL suppressed the translocation of the NF‐κB p65/p50 proteins from the cell cytoplasm to the nucleus and reduced p300 recruitment to the COX‐2 promoter. To further confirm this hypothesis, immunofluorescence assays were performed. As expected, treatment with CS‐6 markedly inhibited translocation of the NF‐κB p65/p50 proteins from cell cytoplasm to nucleus and reduced p300 recruitment by comparison with control group (Figure 6g). The above results show that IATL may inhibit the expression of COX‐2 by inhibiting the translocation of NF‐κB from the cytoplasm to the nucleus and inhibiting the recruitment of p300.

### 3.8 IATL inhibited IKKβ activity in human GBM cells

Previous studies showed that only activated NF‐κB p50/p65 subunits translocate to the nucleus and promote the transcription of target genes.^25^ However, NF‐κB activation depends on the phosphorylation of IκB proteins by the IKK complex. In the canonical pathway, IKKβ is the main upstream kinase and is responsible for the phosphorylation of IκB‐α.^42^ Therefore, we further investigated whether IATL could inhibit IKK activity. As shown in Figure 7a, IATL significantly decreased p‐IκB‐α and p‐IKKβ expression in glioma cells but only mildly suppressed p‐IKKα/β expression. Moreover, using a cell IKKβ kinase activity spectrophotometric quantitative detection kit, we also assessed the inhibition of IKKβ kinase activity by IATL in vitro. As shown in Figure 7b,c, the inhibition of IKKβ kinase activity was similar to that seen in the above experiments. Taken together, these results supported the hypothesis that IATL induced the suppression of NF‐κB/COX‐2 signaling through the inhibition of IKKβ kinase activity.

**Figure 7:** Isoalantolactone (IATL) inhibited IκB kinase β (IKKβ) activity by targeting ATP binding sites. A, After treatment with IATL for 48 h, the expression of IκB‐α, p‐IκB‐α, IKKα/β, and p‐IKKα/β in glioma cells was examined by using Western blotting. (B,C) IKKβ kinase activity in U87 cells was also tested by using the cell IKKβ kinase activity spectrophotometric quantitative assay kit. The activity values and percentages were calculated using the formulas provided. The results are expressed as the means ± SDs of three independent experiments. *P < 0.05, **P < 0.01 vs the dimethyl sulfoxide‐treated group

### 3.9 IATL inhibited the growth of GBM xenografts in nude mice

Based on the in vitro experimental results, we established a GBM *xenograft* nude mouse model to further explore tumor growth inhibition by IATL in vivo. As expected, the tumor volume (Figure 8a) and tumor weight (Figure 8b) were significantly reduced in mice treated with IATL for 14 days compared to the volume and weight of tumors in the control group. The tumor growth inhibition rate in the IATL treatment group (30 mg/kg) was 55.48 ± 12.11% (Figure 8c). No obvious toxic reaction occurred in the mice during treatment. The tumor tissues were harvested for immunohistochemical staining to examine the expression of p‐p65 and COX‐2 in vivo. As shown in Figure 8d, IATL markedly reduced the expression of p‐p65 and COX‐2 in tumor tissue. Taken together, these results indicated that IATL inhibited the growth of *xenograft* human GBM tumors in vivo.

**Figure 8:** Isoalantolactone (IATL) suppressed glioma tumor growth in vivo. The subcutaneous transplant tumor model was established by inoculating U87 cells into nude mice. A, Photographs of tumors from nude mice treated with IATL for 15 d and control‐treated nude mice. (B,C) Tumor volumes and weights were calculated. D, The protein expression of cyclooxygenase 2 and p‐p65 was examined by immunohistochemical analysis (original magnification, 400 × ). E, IATL penetrated the blood‐brain barrier. LC‐MS spectrum of a cerebrospinal fluid sample from the nude mouse model after pretreatment with IATL (1 h)

### 3.10 IATL penetrated the BBB

Most small molecule drugs have difficulty crossing the BBB,^43^ so we performed a puncture assay in mice to collect cerebrospinal fluid for LC‐MS/MS analysis to determine whether IATL could cross the BBB. As shown in Figure 8e, a high peak was detected in the cerebrospinal fluid samples at 2.53 minutes, which was consistent with the peak time for the IATL standard sample. These results implied that IATL could cross the BBB and thus have great potential for the treatment of CNS diseases such as GBM.

## 4 DISCUSSION

Because of the poor clinical outcomes of GBM and the lack of effective chemotherapeutic drugs, finding new targeted therapies is necessary. The natural product IATL has a variety of pharmacological activities; its antitumor activity has been reported, but its role in glioma has not been clarified. However, this study suggested that IATL significantly inhibited GBM growth in a dose‐dependent manner. IATL inhibited the growth of GBM by inhibiting the NF‐κB/COX‐2 signaling pathway and may also induce mitochondrial damage and apoptosis via dephosphorylation and increased mitochondrial translocation of cofilin. In addition, we found here that IATL bound to IKKβ to inhibit the expression of COX‐2 in GBM. IKK is a key regulator in the NF‐κB signaling pathway, and we proved by an in vitro kinase assay that IATL prophylactically inhibits IKK activity (Figure 9).

**Figure 9:** The anticancer mechanism of Isoalantolactone (IATL), with respect to the effect of IATL on IκB kinase β kinase activity, the NF‐κB/cyclooxygenase 2‐mediated signaling cascade, and cofilin translocation‐regulated apoptosis in glioblastoma (GBM)

The overexpression of COX‐2 promotes cell proliferation and increases tumor invasion and migration; thus, COX‐2 plays an important role in tumor development and progression.^44^ In turn, the targeted inhibition of COX‐2 is a potential therapeutic strategy, and finding additional targeted anticancer drugs is important.^45^, ^46^, ^47^, ^48^ Because CB is a classic anti‐inflammatory agent, we used CB as a positive inhibitor of COX‐2 expression. The coadministration of IATL and CB did not further affect the tumor cell death rates, so we hypothesized that IATL exerted its effects through the same molecular mechanism as CB. In addition, the IC_50_ values of IATL in U87 and U251 cells were significantly lower than those of CB, indicating that IATL is more effective than CB as a small molecule inhibitor.

The nuclear transcription factor NF‐κB is involved in the expression of COX‐2 in many cell lines, whereas the transcriptional activity of NF‐κB is influenced by the transcriptional coactivator p300. The transcriptional coactivator p300 can bind to NF‐κB p65/p50 dimers via acetylation or can enhance its own transcriptional activity by modifying the chromatin structure.^49^, ^50^ The current study demonstrated that IATL can inhibit the nuclear translocation of NF‐κB p65/p50 dimers and reduce the recruitment of p300, thereby reducing the binding of these proteins to the COX‐2 promoter region and finally downregulating COX‐2 expression.

The cytoskeleton plays an important regulatory role in the initial stage of apoptosis. The actin depolymerization inhibitor jasplakinolide can stabilize filamentous F‐actin, thereby increasing the activation of caspase‐3. The actin polymerization inhibitor cytochalasin D can also lead to rapid Cyt c release and caspase activation, in turn leading to apoptosis.^51^, ^52^, ^53^ Our laser confocal microscopy and Western blotting results showed that IATL significantly downregulated the expression of filamentous F‐actin and increased the expression of globular G‐actin, indicating the conversion of F‐actin to G‐actin. This change is most likely the reason for the apoptotic effect of IATL on GBM cells. Dephosphorylated cofilin has been reported to undergo mitochondrial translocation, and cofilin phosphorylation inhibits its mitochondrial translocation.^54^, ^55^ The binding of cofilin to actin is a crucial step in apoptosis. Dephosphorylated cofilin is translocated to mitochondria, and its binding to actin induces cytoskeletal remodeling, eventually resulting in the release of mitochondrial Cyt c and ultimately apoptosis.^54^ Because cofilin's mitochondrial translocation is highly dependent on actin's mitochondrial translocation,^55^ exploring the molecular mechanism underlying the mitochondrial translocation of actin and cofilin and the interplay between these proteins is important. Our confocal analysis showed that IATL induced the colocalization of cofilin and globular G‐actin, promoted the colocalization of cofilin and mitochondria, and increased the colocalization of G‐actin and mitochondria. However, no change in the colocalization of F‐actin and mitochondria was found. Furthermore, our immunoprecipitation results indicated that cofilin and actin could directly bind to mitochondria. In summary, we proved that IATL can cause cofilin dephosphorylation, induce cofilin and G‐actin translocation to the mitochondrial inner membrane and thus their mutual binding, and ultimately damage mitochondria to cause apoptosis. In addition, tumor cell migration and invasion are two important factors in metastasis, and the degradation of the extracellular matrix is the key to metastasis. MMP‐2 and MMP‐9 could play an important role in disrupting the extracellular matrix; furthermore, MMP‐2 and MMP‐9 are negatively correlated with the prognosis of glioma patients.^56^, ^57^ Our research also confirmed that IATL significantly reduced the expression of MMP‐2 and MMP‐9 and inhibited the migration and invasion of GBM cells.

The BBB is an important factor that limits the use of chemotherapeutic drugs in the treatment of GBM.^58^ The detection of the concentration of drugs injected into the bloodstream in the cerebrospinal fluid can demonstrate the penetration of the BBB.^59^ We detected IATL in mouse cerebrospinal fluid by LC‐MS/MS analysis, thus demonstrating that IATL can cross the BBB, a necessary occurrence in the treatment of diseases of the CNS.

In conclusion, the current study indicated that IATL effectively inhibited the proliferation of GBM cells and induced apoptosis by inducing cofilin and G‐actin translocation to the mitochondrial inner membrane. Intriguingly, IATL can target the IKKβ cascade signaling pathway and block the NF‐κB signaling pathway. In addition, IATL penetrated the BBB. These findings provide the basis for the clinical use of IATL and provide evidence supporting the further development of potential antitumor drugs.

## CONFLICT OF INTEREST

The authors declare that they have no conflicts of interest.
